# lncRNA SNHG12 Inhibition Based on Microsystem Cell Imaging Technology Protects the Endothelium from LPS-Induced Inflammation by Inhibiting the Expression of miR-140-3p Target Gene fndc5

**DOI:** 10.1155/2022/1681864

**Published:** 2022-08-13

**Authors:** Lei Zhang, Bin Li, Degang Zhang, Ye Zhao, Qin Yu

**Affiliations:** ^1^Department of Critical Care Medicine, The First Hospital of Lanzhou University, The First School of Clinical Medicine of Lanzhou University, Lanzhou 730000, Gansu, China; ^2^Department of Respiratory, Lanzhou University Second Hospital, Lanzhou 730000, China; ^3^The First School of Clinical Medicine of Lanzhou University, The First Hospital of Lanzhou University, Lanzhou 730000, Gansu, China

## Abstract

Acute lung injury (ALI) is a serious disease with a high incidence rate, characterized by uncontrolled inflammation and apoptosis. At present, long-chain noncoding RNA (lncRNA) is a noncoding RNA with a length of more than 200 nucleotides. It plays an important role in ALI, cell cycle regulation, cell differentiation regulation, and many other life activities. Therefore, the current focus is to identify and evaluate the possible functions and potential molecular mechanisms of lncRNA small nuclear host gene 12 (SNHG12). Lipopolysaccharide (LPS)-induced mice model and in vitro cell model were established. Gene knockout is to use the principle of DNA homologous recombination to replace the target gene fragment with the designed homologous fragment, so as to achieve the purpose of gene knockout. The relationship between lncRNA SNHG12 expression and ALI was studied through knockdown and overexpression experiments. The qRT-PCR, ROS, immunohistochemistry, histopathology, TUNEL, and cell permeability tests were performed to further verify the possible targets and mechanisms of action. The expression of lncRNA SNHG12 in lung tissue was lower than that in normal tissue. The results showed that lncRNA SNHG12 could reduce lung cell injury and inflammatory cytokines induced by ALI. Bioinformatics analysis showed that lncRNA SNHG12 interacted with miR-140-3p. Subsequent experiments confirmed the link between lncRNA SNHG12, miR-140-3p, and fndc5. Furthermore, this study indicates that lncRNA SNHG12 has a key function in ALI. The results of this study demonstrated the role of lncRNA SNHG12 in the pathological process of ALI and provided a reference for developing novel anti-ALI treatments so that patients can get timely treatment, avoid causing multiple organ failure, and will not endanger their life safety.

## 1. Introduction

Acute lung injury (ALI) represents various lung disorders causing edema, respiratory failure, and hypoxemia. The clinical symptoms of ALI include declined lung compliance, progressively aggravating hypoxemia, as well as excessive pulmonary inflammation [1]. The causes may be direct lung injury due to severe infection, gastroesophageal reflux, drowning, or indirect injury caused by major burns, extrapulmonary trauma, and massive blood transfusion [2]. In the USA, there are approximately 190,000 new ALI patients diagnosed annually. ALI is usually treated with supportive therapy, accompanied by anti-inflammatory drugs, like antibiotics and glucocorticoids [3]. Additionally, mechanical ventilation has been performed for critical ALI cases that have respiratory failure. However, there have been few reports of specific drugs for ALI. Clinically, the cure rate of ALI is low and the fatality rate is high. Therefore, it is necessary to conduct in-depth research on the pathogenic mechanism of ALI and explore more safe and effective treatment drugs [4].

The incidence rate of ali/ards has been difficult to assess due to regional differences and insufficient overall understanding of the disease. Other factors such as patient age and related clinical diseases also affect the incidence rate of ALI. Clinical factors include sepsis, inhalation, pneumonia, trauma, blood transfusion, pancreatitis, smoke or toxic gas inhalation. Severe sepsis and multiple transfusions are related to the highest incidence of ALI. The lowest rates occur in patients with trauma or drug overdoses. For patients with multiple comorbidities, chronic lung disease, or chronic alcohol abuse, the risk for lung injury is higher [5]. Severe sepsis may lead to sepsis with organ dysfunction such as hypotension, oliguria, lactic acidosis, disturbance of consciousness and abnormal liver and lung functions, which may lead to lung damage and can even be life threatening in severe cases.

lncRNAs, which are transcripts longer than 200 nucleotides and have a limited coding capacity, were once thought to be a waste product of biological metabolism. However, in recent decades, lncRNAs have been discovered to play a role in a distinct biological processes, including cell differentiation, proliferation, apoptosis, and stress responses [2]. lncRNAs have been shown to control gene expression by a variety of mechanisms, including binding to microRNAs, mRNAs, and proteins, as well as epigenetic changes, transcriptional, and posttranscriptional processing. Previous studies have found that some miRNAs can regulate cell differentiation, proliferation, migration, and apoptosis [6]. Presently, the ALI mortality shows a decreasing trend year by year; however, further understanding of the pathogenesis of ALI needs to be deepened due to its high morbidity (about 200,000 cases in the USA annually) and mortality (>35%) [7]. It is well known that changes in miRNA will lead to changes in the molecular expression of targeted genes [8]. Although the abnormal expression of miRNA is usually mild, this mild abnormal expression may lead to huge changes in the expression of target genes, thus having a profound impact on the disease development process [9], while this will thereby impact diverse pathways. Therefore, it has been suggested that suppression of miRNAs can suppress mRNA expression and/or disease-associated gene activities [10].

The lncRNAs have become powerful regulators of many cell processes by interacting with proteins, RNA, and DNA [11]. lncRNAs are associated with a low conservation rate among different species, with lower copy numbers in cells than mRNAs. However, studies have shown that lncRNAs enriched in specific ways in tissues or cells can exert profound phenotypic effects [12]. Li et al. [13] proposed that lncRNAs act as a miR-29b sponge to promote wound healing in diabetic foot ulcers. The functional role and interaction of lncRNA H19, miR-29b, and FBN1 in DFU were then explored by inspecting the proliferation, apoptosis of fibroblasts and migration after silencing H19, inhibiting or overexpressing miR-29b and FBN1. Cheng et al. [14] determined the relationship between long noncoding RNA (lncRNA) H19, mircoRNA29b (miR-29b), and VEGFA in the growth of diabetes mellitus (DM). It was observed that H19 is upregulated and miR-29b downregulated in individuals with DM and directly binds miR-29b. Small nucleolar host gene 12 (SNHG12), which is called LNC04080 as well, can be detected in chromosome 1p35.3, with a full length of 1,867 bases [15]. Four small nucleoli RNAs (SNORA66, SNORA61, SNORA16A, and SNORD99) are encoded by their spliced introns [16]. Studies have shown that lncRNA SNHG12 is associated with many cancers, such as breast cancer, stomach cancer, osteosarcoma, and glioma, as well as other cancer types. Changes in the expression of lncRNA SNHG12 are related to tumor cell growth, viability, invasion, and metastasis, which may also impact cancer patient survival [17]. The lncRNA SNHG12 is upregulated and inhibits tumor inhibition of miRNAs in many cancer types. In addition, lncRNA SNHG12 is also specifically expressed in the intima of progressive or degenerative atherosclerosis, which helps to better understand its potential role and may provide new insights into DNA damage in advanced lesions.

SNHG12, a long noncoding RNA, is involved in a variety of vascular endothelial activities and malignancies. However, the role of lncRNA SNHG12 in ALI is unknown. Therefore, by establishing a mouse ALI model, this study investigated whether lncRNA SNHG12 played a protective role in the process of ALI from the aspects of expression level, inflammatory response, cell permeability, cell apoptosis, target binding test, etc., and explored the effect of lncRNA SNHG12 activation on LPS-induced ALI and its development mechanism at the cellular molecular level. Moreover, this study focused on identifying and evaluating lncRNA SNHG12's role in ALI and revealing the potential molecular mechanism of its role, to provide information for the diagnosis and treatment of ALI.

The remaining sections of the manuscript are organized as follows.  Section 2 is about material and methods in which a detailed description of the proposed experimental process is provided. The results are discussed in Section 3 and Section 4 is the discussion. The conclusion is given in Section 5.

## 2. Materials and Methods

### 2.1. Animals

The BALB/c mice (weight, 18–20 g) belonging to the mammalia class, a mature experimental animal with small size, easy to catch, easy to operate, and with a short growth period, were provided by Shanghai Slack Laboratory Animal Co, Ltd (Shanghai, China). BALB/c is an albino laboratory-bred, immunodeficient house mouse strain from which several common substrains are derived. They are one of the most commonly used inbred strains. All operations were performed under aseptic conditions. Each animal experiment gained approval from the first hospital of Lanzhou University and was performed in line with the guidelines for the Care and Use of Laboratory Animals released via the National Institutes of Health (NIH).

### 2.2. Establishment of the ALI Model

The mice were randomized as a control group (intratracheal infusion with 1.5 mg/kg normal saline), ALI group injected with 3 mg/kg LPS intratracheal (LPS group), LPS + Si-SNHG12 (3 mg/kg LPS + 8 mg/kg Si-SNHG12), and LPS + Si-miR-140-3p (3 mg/kg LPS + 8 mg/kg miR-140-3p) and LPS + NC (3 mg/kg LPS + 2 mg/kg Agomir-NC). At 24 h postinjection of LPS, all animals in each group were euthanized in a CO_2_ chamber, and then the serum was collected, and the expression level was detected by qRT-PCR. The right lung was lavaged with normal saline (0.9%). we harvested bronchoalveolar lavage fluid (BALF) for centrifugation under 4°C (4000 RPM) for 15 mins. Cell granules were collected for cell count determination. BALF supernatant was preserved under 80°C until use. After weighing, we prepared homogenate of left lung tissues with PBS (0.1 mol/L, pH 7.4) on ice. The rest left lung tissues were rinsed by precold saline, followed by 24 h of 10% neutral formaldehyde fixation, to conduct histopathological analysis, Western blotting (WB) analysis, and TUNEL staining.

### 2.3. Quantitative Real-Time PCR Analysis (qRT-PCR)

To analyze miRNAs, we extracted total splenic cellular and lung tissue RNAs with miRNeasy mini kit (QIAGEN) according to specific protocols. Later, stem-loop primers specific to miRNAs (Applied Biosystems, Foster City, CA, USA) were employed for reverse transcription. Afterward, the SYBR Green Master Mixture (Roche) was adopted for the qRT-PCR procedure with the 7500 Fast Real-Time PCR System. SYBR Green qPCR Master Mix (No ROX) is a 2x concentrated, ready-to-use supermix optimized for dye-based quantitative PCR. Sequences of all primers utilized in this experiment were shown below, for si-NC, 5′-UUCUCCGAACGUGUCAC-GUTT-3′ (forward), 5′-ACGUGACACGUUCG-GAGAATT-3 (reverse); and for Si-SNHG12, 5′-GCAGUGUGCUACUGAACUUTT-3′ (forward), 5′-AAGUUCAGUAGCACACUGCTT-3′ (reverse), respectively. GAPDH served as the reference for normalizing mRNA expression. The 2^−ΔΔCt^ approach was adopted for calculating gene expression as described previously [18].

### 2.4. Cell Culture and Transfection

Techniques are used as an analytical tool for determining genetic functioning, protein synthesis, cell growth, and development. In this study, pulmonary microvascular endothelial cells (PMVECs) were cultivated within the RRMI-1640 medium that contained 10% fetal bovine serum (FBS, Gibco, Rockville, MD, USA). FBS provides nutrition, growth, and attachment factors to cells while also protecting them from oxidative damage and apoptosis through mechanisms that are hard to replicate in serum-free medium (SFM) settings. It gives cells in culture a variety of undefined growth-promoting and survival-enhancing factors. When the cell density reached 80%, the inoculation density was 1 : 2. Later, we seeded cells into the six-well plates, followed by transfection using Lipofectamine 2000 (pcDNA US-ing enter-R4000) when the fusion degree was about 60%. Next, 10 *μ*L Lipofectamine 2000 and 10 *μ*L siRNA-SNHG12 were added to a 500 *μ*L serum-free medium, respectively. The dose was 20 nM (pcDNA was prepared from 4 *μ*g EN-Transfer-R4000 and 2.68 *μ*g pcDNA-SNHG12). 1.5 mL 1640 medium (Gibco, Rockville, MD, USA) was added to a Petri dish, equal amounts of Lipofectamine 2000 and sirNA-NC (pcDNA was prepared by Entranster-R4000 and pcDNA-NC) were added into the control group as the experimental group. The medium was replaced 6 h after transfection.

### 2.5. Flow Cytometry

Flow cytometry is one of the most advanced cell quantitative analysis techniques in modern times. It can analyze tens of thousands of cells and measure multiple parameters from a cell at the same time. In flow cytometry single or several lasers are used to enable a multiparametric examination of single cells. In this study cells were harvested to detect cell apoptosis. In brief, the collected cells were subject to FITC-Annexin V/propidium iodide (PI) staining according to FITC Annexin V Apoptosis Detection Kit (BD Biosciences, USA) instructions. Later, we used the prechilled 75% ethanol to fix cells for a 24 h period before analysis.

### 2.6. Transwell Assay

The Transwell Assay is also known as the Boyden or modified Boyden chamber assay. PMVECs in diverse groups were classified as 1 × 10^5^ cells/chamber were inoculated into Transwell chambers (Corning costar, Corning, New York, USA), followed by a 72 h culture. Afterward, the original medium was discarded, upper chamber cells were incubated with the 1 mg/ml FITC-dextran (200 *μ*l, molecular weight 4000; Sigma; Cat No. 46944) for a 15-min period under 37°C. Thereafter, the fluorescent microplate reader (m200 pro, TECAN, Switzerland) was employed to detect dye intensity within the bottom chamber at 485 nm. Each assay was carried out thrice.

### 2.7. ELISA

An enzyme-linked immunosorbent assay (ELISA) or enzyme-linked immunosorbent assay (EIA) is a blood test that identifies and quantifies antibodies. This test can be used to determine antibodies specific to infectious diseases. ELISA kits (Elabscience Biotechnology Co., LTD., Wuhan, China) were adopted to determine TNF-*α*, IL-1*β*, and IL-6 protein expression in cells and BALF in line with specific protocols. All samples were carried out thrice independently.

### 2.8. Luciferase Assay

A luciferase assay is used to determine if a protein can activate or repress the expression of a target gene. When achieving 60–70% confluence, microRNA-miR-140-3p mimic was cotransfected with pMicroRNA-Reporter-SNHG12-WT or pMicroRNA-reporter-SNHG12-MUT into cells.

Lipofectamine 2000 (Carls bad Invitrogen, California, USA) was used to provide high transfection efficiency and activity.

The luciferase was detected in the treated cells through a dual-luciferase reporter assay (Promega, MAD-ISON, WI, USA).

### 2.9. Histopathologic Analysis

Histopathology is the microscopic examination of a biopsy or surgical specimen that has been processed and put onto glass slides to determine the signs of disease. For assessing lung injury, we collected mouse left lung tissues at 24 h postinjection of LPS. Later, the tissues were subject to 4% (V/V) paraformaldehyde fixation, paraffin embedding, slicing into 4-*μ*m sections, and HE (Sigma-Aldrich) staining. Finally, sections were monitored with a microscope. We rated the histological changes according to Eveillard, Soltner, and Parsey MV's classical lung injury score [18, 19].

### 2.10. Determination of Reactive Oxygen Species

We grew cells (2 × 10^5^/well) into the plates. To be specific, cells were pretreated with aloin at varying concentrations (100, 150, 200 *μ*g/ml) under 37°C and exposed to LPS for a 30 min period. Then, the Reactive Oxygen Species (ROS) Assay kit (Beyotime Institute of Biotechnology) was utilized to detect total ROS levels in cells in line with specific instructions. In brief, we removed the original medium and added dichloro-dihydro-fluorescein diacetate (DCFH-DA) (final concentration, 10 *μ*M) to incubate cells for a 20 min period under 5% CO_2_ and 37°C conditions. The inverted fluorescence microscope (Olympus Corporation, Tokyo, Japan; magnification, 100x) was utilized to observe ROS levels, whereas Image J software (version 1.46, National Institutes of Health, Bethesda, MD, USA) was adopted for quantitation. Each experiment was repeated thrice.

### 2.11. Immunohistochemistry (IHC)

Immunohistochemistry (IHC) is a technique for determining the tissue distribution of an antigen of interest in health and disease using monoclonal and polyclonal antibodies. Specific tumor antigens are expressed de novo or upregulated in particular tumors, and IHC is commonly utilized for cancer diagnosis. In this study, the slices were soaked in xylene for 15 min before being rehydrated with gradient ethanol. Thereafter, citric acid (pH 6.0 DAKO) was utilized to incubate sections for a 10-min period. When cooling to ambient temperature, we rinsed sections with water and PBS for a 15-min period and later incubated those using 3% H_2_O_2_ for a 10-min period. After blocking for a 30-min period using 5% bovine serum albumin (BSA), a primary antibody was utilized to incubate sections overnight under 4°C, followed by developing a DAB color-rendering kit (Soleibol). A panoramic scanning electron microscope was used to scan the sections and observe the images.

### 2.12. Western Blotting (WB) Assay

It is a common method for detecting a specific protein in a complicated matrix-like cell or tissue lysate (i.e. protein extracts). The Western blot technique separates proteins by molecular weight using gel electrophoresis (SDS-PAGE or native PAGE). WB assay was performed to detect CD31 expression. Briefly, 10% SDS-PAGE was conducted to separate proteins (25 *μ*g per sample), followed by transfer onto PVDF membranes (Millipore, Billerica, MA, USA). Later, 5% nonfat milk in TBST was used to block membranes. Thereafter, the anti-CD31 primary antibody (1 : 5000, Abcam, Shanghai, China) was used to incubate protein blots under 4°C overnight, followed by incubation using HRP-labeled secondary antibody (1 : 10000, Solarbio, Beijing, China). Finally, results were visualized using the chemiluminescence detection system (Millipore, Billerica, MA, USA), whereas Quantity One software (Bio-Rad, Hercules, CA, USA) was employed for band quantitation.

### 2.13. TUNEL Staining

TUNEL staining (terminal deoxynucleotidyl transferase dUTP Nick end labeling), also known as the TUNEL assay, detects DNA breaks caused by DNA fragmentation during apoptosis' final phase. DUTP can connect to the 3′-oh terminal of DNA broken in apoptotic cells under the action of deoxyribonucleotide terminal transfer, and accurately detect apoptotic cells through chemical color development. The lung tissue sections were dewaxed with xylene, followed by gradient ethanol rehydration (100%–70%, V/V), and rinsing with water. 100 *μ*L protease K (20 *μ*g/ml, Roche) was treated under ambient temperature for a 15-min period and rinsed by PBS thrice. Cells were later stained with freshly prepared TUNEL solution by adopting the TUNEL apoptosis assay kit (ALexa Fluor 488) (Roche, Basel, Switzerland). Later, three fields of view (FOVs) were chosen from every section to count the TUNEL-positive cells under the inverted fluorescence microscope (DP73; Olympus; magnification, 400x).

### 2.14. Statistical Analysis

Results were presented in the form of means ± SD. Comparison of two groups was conducted by Student's *t*-test, and one-way analysis of variance (ANOVA) was employed to analyze differences across multiple groups. GraphPad Prim 5 (GraphPad Software, La Jolla, CA, USA) was employed for statistical analysis. *P* < 0.05 indicated statistical significance.

## 3. Results

### 3.1. lncRNA SNHG12 Was Downregulated in LPS-Induced ALI

Low expression of SNHG12 in lung tissue samples of LPS-induced ALI mice was detected by qRT-PCR (Figures 1(a) and 1(b)). Meanwhile, ELISA was conducted to detect inflammatory cytokine levels within BAL. As a result, those within the ALI group markedly increased relative to the control group as shown in Figure 1(c).

### 3.2. SNHG12 Ameliorates Lung Endothelial Cell Injury

We first detected the level of SNHG12 in PMVECs cells by qRT-PCR. As a result, the intracellular SNHG12 expression remarkably elevated posttransfection of the overexpressed plasmid (Figures 2(a) and 2(b)). The detection of apoptosis level showed that SH could effectively reduce lPS-induced apoptosis as shown in Figure 2(c). Moreover, based on the results, LPS dramatically elevated proinflammatory cytokine contents, like IL-1*β*, TNF-*α*, and IL-6 within ALI relative to control, while SNHG12 treatment suppressed proinflammatory cytokine levels induced by LPS (Figure 2(d)). Furthermore, LPS elevated cell permeability and ROS levels relative to control, whereas SNHG12 significantly inhibited ROS and cell permeability (Figures 2(e) and 2(f)). Based on the above results, SNHG12 may be involved in the biological process of ALI, which will be further explored in subsequent studies.

### 3.3. The Target of SNHG12 Was Predicted and Validated

According to Figure 3(a), SNHG12's complementary sequence could be detected within 5′-UTR in miR-140-3p. Besides, as revealed by the luciferase reporter gene assay, SNHG12 and miR-140-3p could interact with each other (Figure 3(b)). Moreover, the miR-140-3p mRNA expression remarkably decreased after overexpression of miR-140-3p (Figure 3(c)). Based on flow cytometry, miR-140-3p could further reduce the lPS-induced apoptosis that had been alleviated by SNHG12 (Figure 3(d)). Furthermore, SNHG12 suppression remarkably elevated proinflammatory cytokine levels relative to the LPS-induced group, whereas miR-140-3p treatment showed partial reduction (Figure 3(e)). Additionally, miR-140-3p treatment can partially downregulate the ROS and cell permeability levels (Figures 3(f) and 3(g)).

### 3.4. fndc5 was a Direct Target of miR-140-3p

The potential targets of the miR-140-3p were predicated. The results showed that the fndc5 was considered as one of the candidates after analysis. We discovered miR-140-3p′s sequence within 3′-UTR in fndc5 (Figure 4(a)). In addition, it was verified through luciferase reporter gene assay that miR-140-3p is bound to fndc5 (Figure 4(b)). Moreover, fndc5 mRNA expression remarkably decreased when miR-140-3p was overexpressed (Figure 4(c)). Besides, the simultaneous upregulation of fndc5 and miR-140-3p could more effectively reduce apoptosis (Figure 4(d)). Furthermore, relative to the LPS-induced group, the overexpression of miR-140-3p significantly increased the levels of proinflammatory cytokines, ROS, and cell permeability. However, fndc5 treatment partially downregulates these levels (Figures 4(e)–4(g)).

### 3.5. SNHG12 Could Alleviate LPS-Induced ALI in Mice

To determine whether SNHG12 alleviates LPS-induced ALI in mice, we first detected the levels of SNHG12, miR-140-3p, and fndc5. The results showed that the levels of SNHG12 and fndc5 among mice treated with LPS declined, while the levels of MI-140-3p were increased (Figure 5(a)).

Histological analysis showed that SNHG12 reduced the degree of pulmonary lesions and reduced lesion distribution relative to the LPS group. The TUNEL staining test showed that LPS elevated TUNEL-positive cell numbers relative to control, whereas SNHG12 injection had the opposite effect. Meanwhile, SNHG12 treatment markedly suppressed the proinflammatory cytokine levels within BALF induced by LPS. As revealed by WB assay, the fluorescence intensity of the LPS-induced group decreased relative to control, while the fluorescence intensity of the SNHG12 treatment group increased, suggesting that SNHG12 could improve fibrosis and alleviate LPS-induced ALI in mice.

## 4. Discussion

So far, the role of lncRNA SNHG12 in ALI is still unclear. Our results showed that lncRNA SNHG12 was downregulated in lung tissue compared with normal lung tissue, suggesting that lncRNA SNHG12 may be a biomarker for predicting ALI. In addition, overexpression of lncRNA SNHG12 significantly reduced the apoptosis index (TUNEL-positive cells) in ALI mice. The results showed that lncRNA SNHG12 played a key role in the occurrence and development of ALI on the basis of improving lung endothelial injury. To sum up, these results implied that lncRNA SNHG12 protected against ALI through suppressing apoptosis, confirming that lncRNA expression is unregulated in various physiological and pathological processes [20, 21] and has a certain function in disease occurrence [22–24]. However, a detailed explanation requires further research to prove the relationship between lncRNA SNHG12 and ALI.

Inflammatory response exerts a key function in initiating and maintaining ALI [25]. Reducing the level of plasma inflammatory factors and the pathological damage of lung tissue can play a role in the treatment of ALI [26]. Proinflammatory cytokines such as IL-1*β*, IL-6, and TNF-*α* increase the permeability of lung epithelial cells, further causing damage to lung tissues as well as neutrophil accumulation, resulting in pulmonary edema [27]. Il-6 expression increases within BALF of ALI cases, while a high level of IL-6 increases mortality, which has been suggested to be the monitoring biomarker for ALI [28]. In the present study, the results showed that lncRNA SNHG12 reduces proinflammatory cytokines such as IL-1*β*, IL-6, and TNF-*α* in BALF. These results suggest that lncRNA SNHG12 improves intrapulmonary ALI and inhibits inflammatory responses.

Studying the cross-talk between lncRNA and miRNA helps to understand the pathogenic mechanism underlying ALI [29]. As revealed by recent research, miRNAs control gene levels during the critical ALI processes [30, 31]. According to the results of this study, lncRNA SNHG12 regulates ALI by targeting miR-140-3p. First, we conducted bioinformatics analysis, and the results showed that lncRNA SNHG12 might interact with miR-140-3p. Subsequently, we confirmed the combination of miR-140-3p with lncRNA SNHG12 through a dual-luciferase assay. In addition, qRT-PCR revealed that, miR-140-3p expression in ALI cells elevated within LPS-mediated ALI, and that miR-140-3p endogenously interacted with lncRNA SNHG12. According to permeability and ROS analysis, lncRNA SNHG12 interacted with miR-140-3p. Finally, miR-140-3p overexpression decreased inflammatory factor expression following RNA knockdown. Collectively, such findings indicated the role of lncRNA SNHG12 in regulating miR-140-3p of the target gene as an endogenous sponge or ceRNA. The expression of lncRNA pacer in alveolar macrophages of ALI patients and lung tissues of ALI mice was significantly increased; after overexpression of pacer, tumor necrosis factor-*α* (TNF-*α*) the expression of TNF was increased, while after knockdown of pacer, the inflammatory factor TNF-*α*,the expression of IL-6 decreased; TNF in lung tissue and serum of ALI mice after pacer knockdown-*α*, the expression of IL-6 decreased significantly, and the degree of lung injury decreased significantly.

For a better understanding of the mechanism underlying miR-140-3p, we performed a bioinformatics analysis. The results revealed fndc5 as miR-140-3p′s putative target. fndc5 is a novel player in metabolic physiology and pathology [32]. In this study, we found that overexpression of fndc5 decreased the effect of miR-140-3p on promoting inflammatory response and apoptosis. In addition, according to qRT-PCR results, miR-140-3p over-expression was related to fndc5 expression. Based on the above findings, miR-140-3p affected inflammatory response in ALI by regulating the fndc5.

## 5. Conclusion

The lncRNAs are a new class of noncoding RNAs that play a crucial role in gene expression in multicellular organisms' growth. Increasing data suggest that lncRNAs play an important role in biological processes like cell proliferation and apoptosis. This study suggests that lncRNA SNHG12 may play a critical part in ALI occurrence, which is the potential molecular target for the diagnosis and treatment of ALI. In addition, by accurately targeting a certain target of cells, it can avoid relatively small damage to normal cells, improve the therapeutic effect, and be highly selective. We found that lncRNA SNHG12 plays a role in the ALI process via modulating miR-140-3p/fndc5 pathway. Therefore, the present work identified and evaluated lncRNA small nuclear host gene 12 (SNHG12) possible function as well as the underlying molecular mechanisms. LPS-induced mice model and in vitro cell model were developed. The relationship between lncRNA SNHG12 expression and ALI was studied through knockdown and overexpression experiments. Subsequent experiments validated the relationship between lncRNA SNHG12, miR-140-3p, and fndc5. This study showed that lncRNA SNHG12 has an important role in ALI. The results of this study confirmed the role of lncRNA SNHG12 in the pathological process of ALI and provided a reference for developing novel anti-ALI treatments.

## Figures and Tables

**Figure 1:** lncRNA SNHG12 was downregulated in LPS-induced ALI. Low expression of SNHG12 in lung tissue samples of ALI mice was detected by qRT-PCR (a, b). Inflammatory cytokine expression levels within BALF were detected by ELISA, and the levels of inflammatory cytokines in ALI remarkably increased compared with the control group (c). ^*∗∗*^*P* < 0.01; ^*∗∗∗*^*P* < 0.001.

**Figure 2:** SNHG12 ameliorates lung endothelial cell injury. The overexpressed SNHG12 vector was constructed, and the overexpressed SNHG12 was selected from PMVEC cell lines. After cell transfection, the overexpression effect was verified by qRT-PCR (a, b). Flow cytometry was conducted to analyze apoptosis levels (c). TNF-*α*, IL-1*β*, and IL-6 expression was analyzed via ELISA (d). ROS levels were detected by ROS kits (e). The cell permeability experiment was performed (f). ^*∗∗*^*P* < 0.01; ^*∗∗∗*^*P* < 0.001.

**Figure 3:** SNHG12 target validation. LncBASE2.1 was used to predict binding targets (a), while the interaction was verified through luciferase reporter gene assay (b). The result of qRT-PCR showed the expression level of miR-140-3p (c). Apoptosis level was detected by flow cytometry (d). In addition, ELISA was used to detect inflammatory cytokines in cell supernatant (e). ROS levels were detected by ROS kits (f). Finally, the cell permeability experiment was performed (g). ^*∗∗*^*P* < 0.01; ^*∗∗∗*^*P* < 0.001.

**Figure 4:** The downstream target of miR-140-3p is fndc5. fndc5 was estimated as miR-140-3p′s target (a). Luciferase report confirmed the targeted combination of fndc5 and miR-140-3p and the direct interaction between the two molecules (b). The fndc5 level was detected by qRT-PCR (c). Apoptosis level was detected by flow cytometry (d). Inflammatory cytokine expression within supernatant was analyzed via ELISA (e). ROS levels were detected (f). Cell permeability test (g). ^*∗∗*^*P* < 0.01; ^*∗∗∗*^*P* < 0.001.

**Figure 5:** SNHG12 alleviates lung injury. SNHG12, fndc5, and miR-140-3p expression were analyzed via qRT-PCR after tail vein injection of SNHG12 (a). H&E staining of lung tissue (b). Tissue TUNEL staining and statistics (c). Inflammatory cytokines in BALF were detected by ELISA (d). The expression of CD31 was determined by Western blot (e). ^*∗∗*^*P* < 0.01; ^*∗∗∗*^*P* < 0.001.

## Data Availability

The data underlying the results presented in the study are included within the manuscript.
